# MtDNA genetic diversity and structure of Eurasian Collared Dove (*Streptopelia decaocto*)

This article has been retracted.

**DOI:** 10.1371/journal.pone.0193935

**Published:** 2018-03-08

**Authors:** Zoltán Bagi, Evangelos Antonis Dimopoulos, Dimitrios Loukovitis, Cyril Eraud, Szilvia Kusza

**Affiliations:** 1 Animal Genetic Laboratory, University of Debrecen, Debrecen, Hungary; 2 Department of Genetics, Development and Molecular Biology, Aristotle University of Thessaloniki, Thessaloniki, Greece; 3 Lab of Agrobiotechnology and Inspection of Agricultural Products, Alexander Technological Educational Institute of Thessaloniki, Thessaloniki, Greece; 4 Unité Avifaune migratrice, Office National de la Chasse et de la Faune Sauvage, Villiers-en-Bois, France; National Cheng Kung University, TAIWAN

## Abstract

The Eurasian Collared Dove (*Streptopelia decaocto*) is one of the most successful biological invaders among terrestrial vertebrates. However, little information is available on the genetic diversity of the species. A total of 134 Eurasian Collared Doves from Europe, Asia and the Caribbean (n = 20) were studied by sequencing a 658-bp length of mitochondrial DNA (mtDNA) cytochrome oxidase I (COI). Fifty-two different haplotypes and relatively high haplotype and nucleotide diversities (H*d*±SD = 0.843±0.037 and π±SD = 0.026±0.013) were detected. Haplotype Ht1 was particularly dominant: it included 44.03% of the studied individuals, and contained sequences from 75% of the studied countries. Various analyses (F_ST_, AMOVA, STRUCTURE) distinguished 2 groups on the genetic level, designated ‘A’ and ‘B’. Two groups were also separated in the median-joining network and the maximum likelihood tree. The results of the neutrality tests were negative (Fu *F*_*S*_ = -25.914; Tajima *D* = -2.606) and significantly different from zero (*P*≤0.001) for group A, whereas both values for group B were positive (Fu *F*_*S*_ = 1.811; Tajima *D =* 0.674) and not significant (*P*>0.05). Statistically significant positive autocorrelation was revealed among individuals located up to 2000 km apart (r = 0.124; P = 0.001). The present results provide the first information on the genetic diversity and structure of the Eurasian Collared Dove, and can thereby serve as a factual and comparative basis for similar studies in the future.

## Introduction

The Eurasian Collared Dove (*Streptopelia decaocto*) is one of the most successful biological invaders among terrestrial vertebrates [1]. The Eurasian Collared Dove began its expansion from India in the sixteenth century and has colonised major parts of Europe, the Middle East, the Caribbean islands and Asia throughout the centuries [2–5]. It reached North Africa in the late 1980s and its spread is still continuing [6–7]. North America and Australia were colonised with human assistance [8–9]. Colonisation of Europe has occurred in the last 50–60 years [10–13], where the present breeding population is estimated to number 7,910,000–14,300,000 breeding pairs, equivalent to 24,100,000–43,000,000 individuals. Europe represents ca. 40% of the global range; the estimated population size is 60,000,000–110,000,000 individuals and the distribution area is 93,400,000 km^2^ [14].

So far ecological studies have been performed on the species mainly with a special focus on the patterns of its expansion, the background of its successful invasion and the impacts of newcomers in the indigenous communities [4, 12, 13, 15, 16]. Several factors have been mentioned as causes of the spread, namely: genetic alteration; emigration unrelated to population density; high adaptability to human habitation; broad diet; and high reproductive output [9].

Although the species attracts wide scientific interest, very little is known about its genetic diversity and structure. In spite of the fact that genetic studies may reveal such elements of the expansion that would be hidden if only classical ornithological methods are used (e.g. source populations, dispersal paths, hidden expansion waves). Expansion can be caused by genetic change in the peripheral area of the species' geographical range [15,17]. Already in 1993 a genetic study on the peripheral populations of the Eurasian Collared Dove was suggested, in order to understand if on the vast and ecologically varied sub-continent of North America such differentiation could take place [15]. Johnson et al. [18] were the first to perform a study on the phylogenetic relationships of the dove genus *Streptopelia* in 2001. They used both nuclear and mitochondrial genes: cytochrome-b (cytb), cytochrome oxidase I (COI), NADH dehydrogenase subunit 2 (ND2) and the nuclear gene β-fibrinogen intron 7 (FIB7). Despite the lower homoplasmy presented in the FIB7 sequences, mitochondrial genes provided better resolution for the phylogeny of *Streptopelia*. Other barcoding and phylogenetic studies were later also carried out mostly in the COI region [19–23].

Here we present the results of the first large-scale study on the variability of the mitochondrial COI region in Eurasian Collared Doves from Europe, Asia and the Caribbean. We determined the level of genetic variability, the demographic events and the possible structuring of the populations, and looked for association between genetic similarity and geographical distance.

## Materials and methods

### Sampling, DNA extraction and sequencing

Samples (n = 134) were collected from altogether 14 countries between 2013 and 2015 (Fig 1, Table 1, S1 Table). In the course of sampling, we were careful to ensure the statistical independence of the samples. A single sample was used from each sampling point (in the case of feathers and eggshells, a sampling point means one nesting or resting place; in the case of tissue it means a road section or an agricultural area, etc.). Moulted feathers on the ground are strongly degraded within a relatively short time (a few months); for this reason, only intact or slightly damaged feathers, left by the doves no more than a few weeks before collection were used. Feathers were stored at room temperature in a dark, dry place between arrival and DNA extraction. Primary and secondary feathers were preferred, since–due to their bigger *calamus* size–the Eurasian Collared Dove’s feathers do not contain enough blood for the extraction method used in the study. Muscle tissues and eggshells were stored in Eppendorf tubes filled with 96% ethanol at -20°C.

**Fig 1:** Populations assigned for examination of divergence between populations.

**Table 1:** Sample size (n), total number of haplotypes (Ht), number of polymorphisms (NP), haplotype diversity (H*d*± SD) and nucleotide diversity (π ± SD) observed in *S*. *decaocto*.

Groups Indices	n	Ht	NP	H*d* ± SD	π ± SD
**Pop1**	6	3	67	0.7333±0.155	0.035±0.021
**Pop2**	5	4	6	0.900±0.161	0.004±0.003
**Pop3**	7	4	3	0.810±0.130	0.002±0.002
**Pop4**	10	7	78	0.867±0.107	0.042±0.022
**Pop5**	7	5	76	0.905±0.103	0.054±0.031
**Pop6**	24	14	79	0.899±0.048	0.012±0.006
**Pop7**	10	10	73	1.000±0.045	0.025±0.014
**Pop8**	6	4	7	0.800±0.172	0.004±0.003
**Pop9**	8	7	113	0.964±0.077	0.065±0.036
**Pop10**	3	2	68	0.667±0.314	0.069±0.052
**Pop11**	4	1	0	0.000±0.000	0.000±0.000
**Pop12**	11	7	83	0.909±0.066	0.025±0.013
**Pop13**	10	7	86	0.867±0.107	0.044±0.024
**Pop14**	12	8	29	0.845±0.104	0.010±0.010
**Pop15**	11	4	82	0.491±0.175	0.024±0.013
**Western Europe**	37	20	111	0.836±0.061	0.023±0.012
**Central Europe**	78	33	118	0.871±0.035	0.023±0.012
**South-Eastern Europe**	8	7	113	0.964±0.077	0.064±0.036
**Caribbean**	11	4	82	0.491±0.175	0.024±0.013
**Group A**	120	42	93	0.804±0.037	0.006±0.003
**Group B**	14	10	62	0.945±0.045	0.034±0.018
**All samples**	134	52	171	0.843±0.037	0.026±0.013

DNA was extracted from feathers (n = 86) using a special method developed by Vili [24], and from tissues (n = 45) and eggshells (n = 3) by the GeneJET Genomic DNA Purification Kit (Thermo Scientific, USA).

Amplification of the 749 bp fragment of the mitochondrial DNA COI was performed using the following primer pairs [23] forward: 5'-TTCTCCAACCACAAAGACATTGGCAC-3'; reverse: 5'-ACGTGGGAGATAATTCCAAATCCTG-3'. The 10 μl reaction volume contained 1 μl dNTP (2 mM), (Thermo Scientific, USA), 2 μl buffer (5 u/μl) (Promega, USA), 2 μl MgCl_2_ (2 mM) (Promega, USA), 0.4 μl primer (10 pmol/μl) (Sigma, USA), 0.2 μl GoTaq polymerase (1.25 U) (Promega, USA), 2.4 μl dH_2_O and 2 μl DNS template.

PCR reaction conditions were the following: 94°C for 5 minutes, then for 35 cycles: 94°C for 1 minute, 60°C for 1 minute, 72°C for 1 minute, followed by 72°C for 5 minutes. PCR products were checked under UV illumination and, if considered useable, prepared for sequencing. Prepared samples were stored at -20°C until sequencing. Sequencing was performed by Macrogen Europe Laboratory in the Netherlands.

### Ethics statement

Moulted primary feathers (n = 86) were collected, but muscle tissue (n = 45) and hatched eggshells (n = 3) were also collected. Sampling of moulted feathers and eggshells is considered as a non-invasive method, which meets the standards of science ethics and does not require special permits. Feather samples from the different countries were obtained from collaborating ornithologists, and were used with their permission. Fresh muscle tissues were sampled only in Hungary from legally hunted unprotected Eurasian Collared Doves or from individuals hit by cars on roadsides. Animals were not shot only for the purpose of this study. No ethics statement was required. Hunters collected samples in accordance with Hungarian national regulations on Eurasian Collared Dove management (decree: 79/2004. (V. 4.) FVM rendelet a vad védelméről, a vadgazdálkodásról, valamint a vadászatról szóló 1996. évi LV. törvény végrehajtásának szabályairól https://net.jogtar.hu/jr/gen/hjegy_doc.cgi?docid=a0400079.fvm).

### Data analysis

Sequences were checked by MEGA6 [25]; problems, if any, were manually corrected. The dividing of sequences was done by CLUSTALW [26]. MEGA6 software was used for fitting the sequences into equal fragments (658 bp). We hypothesized that there are genetic differences between the examined individuals based on geographical location, therefore groups were assigned (n = 15 and n = 4) to contain approximately equal numbers of individuals each (Fig 1). For each group and subsequently for 4 larger geographical areas, diversity indexes (total number of haplotypes (Ht), haplotype diversity (H*d*) and nucleotide diversity (π)) were determined by ARLEQUIN 3.5.2. software [27]. The whole mitochondrial genome of *Streptopelia decaocto* (GenBank: KX372273) was used as a reference sequence for the determination of variable positions. All the available Eurasian Collared Dove sequences (n = 18, S1 Table) derived from the NCBI gene bank and were involved in data analysis. A median-joining network was constructed for all 152 sequences using Network 4.6 [28], in order to establish the overall pattern of the mitochondrial genetic variation of *S*. *decaocto*.

An analysis of molecular variance (AMOVA) [29–30] was performed to estimate the hierarchical genetic structure of each population. Genetic variances were partitioned between populations and within populations. F_ST_s for genetic and geographic groups were calculated and their deviations from zero were tested to estimate the extent of genetic differentiation among populations with the ARLEQUIN 3.5.2. software [27]. The bootstrap consensus tree describing the genetic distances of COI haplotypes was constructed by MEGA6 [25] software with the HKY-model-based Maximum Likelihood method [31] and implemented 1000 bootstrap repetitions [32]. *Phasianus colchicus* (JN850750.1) was used as outgroup.

Population structure and the most likely genetic classification were determined using the admixture model of the STRUCTURE 2.3.4 software [33], which compares the allele patterns of the individuals in pairs and assigns genotypes to groups without pre-hypothesis. To identify the number of clusters (K) that best explained the data, we calculated the rate of change of L(K) (ΔK) between successive K values, as shown by Evanno [34]. In the present study the MCMC algorithm was used in 100 000 repetitions in addition to 10 000 burn-in steps, and 10 iterations were set up for each different K value (K = number of groups). The results of the STRUCTURE analysis were processed by HARVESTER [35]. Three tests of ARLEQUIN 3.5.2. software [27] were applied to test the recent population expansion: Fu’s *Fs* [36], Tajima's *D* [37] and the mismatch distribution using the sum of squared deviations *SSD* [38] and Harpending’s raggedness index (r) [39] with significance inferred using 1000 bootstrap replicates.

Spatial autocorrelation analysis was performed using GenAlEx 6.501 software [40, 41]. This analysis uses a multilocus genetic distance measure [42] that strengthens the spatial signal by reducing locus-to-locus and allele-to-allele variability. The autocorrelation coefficient r is a measure of the genetic similarity between individuals that fall within a defined distance class. The significance of r is determined by random permutation of all individuals among distance classes and recalculating r 1000 times to set the upper and lower 95% confidence limits around this value. In those cases when the value of r fell above or below these limits, significant spatial structure was inferred. 95% confidence intervals were also calculated around each r value by bootstrapping r values within each distance class 1000 times. When these 95% confidence values did not include r = 0, significant spatial structure was inferred. These values also provided a graphical test of significance among r values in different distance classes. Due to the haploid feature of the data, it was not possible to assign the populations with high certainty, therefore the process by Williams [43] was applied in the course of spatial structure analysis, making haploid data applicable in the examination. The point of the process is that all samples are treated as a single population during spatial structure analysis.

## Results

Based on the 658 bp mitochondrial DNA COI sequence of 134 animals, 171 polymorphisms and 52 haplotypes were identified (Table 1). All haplotypes were deposited to GenBank (accession numbers MF381956 –MF382007). Five of these (Ht32, Ht1, Ht47, Ht5 and Ht21) were identical to haplotypes detected earlier [20–23, 44], whereas 47 have not been detected previously and were not geographically restricted. Thirty-seven haplotypes were singletons. Both haplotype and nucleotide diversity were relatively high (0.843±0.037 and 0.026±0.013, respectively) (Table 1). In consideration of the created population based on their geographical localisation, the highest haplotype diversity (1.000) was measured in the Western Hungarian population (Pop7) and the lowest in the Dutch population (Pop11). In the case of other populations, both haplotype diversity and nucleotide diversity were heterogeneous, ranging between 0.491±0.175 (Pop15) and 0.964±0.077 (Pop9), and between 0.002±0.002 (Pop3) and 0.069±0.052 (Pop10), respectively. When we studied the larger geographical regions, 7 haplotypes and 117 polymorphisms were detected in South-Eastern Europe with the highest haplotype and nucleotide diversity (0.964±0.036 and 0.064±0.036). In Central Europe the presence of 33 haplotypes, 118 polymorphisms, a haplotype diversity of 0.871±0.035 and a nucleotide diversity of 0.023±0.012 were detected. In Western European populations 20 haplotypes and 111 polymorphisms were found. Haplotype diversity was 0.836±0.061, and nucleotide diversity was 0.023±0.012. The Caribbean population yielded 82 polymorphisms in addition to 4 haplotypes with low haplotype and nucleotide diversity (0.491±0.175 and 0.024 ±0.013) (Table 1).

A haplotype network was created from data of the present study and 18 Genbank mtDNA COI sequences (Fig 2). Ht1, which was found in 83 individuals proved to be the most frequent haplotype, followed by Ht2 (14 individuals in 6 populations) and Ht3 (10 individuals in 2 populations). Ht1 occurred in 75% of the countries where samples originated from, and it is the most likely common ancestor. The pattern of the network revealed two main groups designated ‘A’ (42 haplotypes found in 120 samples, Table 1) and ‘B’ (10 haplotypes found in 14 samples, Table 1), but did not indicate any clear phylogeographic pattern, and both groups were widely distributed throughout the area studied. The haplotype network for group ‘A’ showed a star-like phylogeny, with most of the haplotypes closely related to the common central haplotype (Ht1), which suggests population expansion. No dominant haplotype and star-like topology were observed in group ‘B’.

**Fig 2:** Median-joining network based on the joint data set (present and GenBank sequences) from mtDNA COI region of *Streptopelia decaocto*. The Figure contains original as well as published sequences. Each circle represents a haplotype with the size proportional to the frequency of collapsed sequences. Solid branches connecting circles represent nucleotide changes among haplotypes. Numbers on branches represent the number of mutational steps between haplotypes. Absence of numbers is equivalent to a single mutational event. Colours and patterns within circles illustrate the relative frequencies of sequences from different geographic areas.

In addition to the haplotype network tree, a phylogenetic tree (Fig 3) provided further confirmation of existence of the two groups among our haplotypes. The separation of the two genetic clusters is also apparent on the Maximum Likelihood Tree (Fig 3).

**Fig 3:** Maximum likelihood bootstrap tree phylogeny based on the joint (present and Genbank sequences) data set from the mtDNA COI region of *Streptopelia decaocto*. Numbers above the branches refer to NJ bootstrap values. Brackets highlight the two genetic groups. *Phasianus colchicus* (JN850750.1) was used as outgroup.

AMOVA results based on the 4 large geographically differentiated populations indicated that genetic variation clearly appeared within populations (98.550%), which can support the weak geographical genetic structure in our samples. However, the analysis based on the two newly described groups gave the opposite result (91.27% variation between the two groups, 8.75% variation within populations, average F_ST_ = 0.912, p = 0.000), and indicated strong genetic differentiations between groups ‘A’ and ‘B’. Variation within (98.70%) and among populations (1.3%) was also analysed for all samples as one group (Table 2).

**Table 2:** Analysis of molecular variance (AMOVA) for populations of *Streptopelia decaocto* based on data from COI loci.

Source of variation	df	Sum of squares	Variance components	% of variation	F-statistics	*p* value
**Geographically based grouping (Western-, Central-, South-East Europe and Caribbean)**						
**Between groups**	3	30.249	0.035	0.420	F_ST_: 0.010	0.007
**Between regions within groups**	11	99.363	0.087	1.000	F_SC_: 0.015	0.000
**Within populations**	9	988.089	8.303	98.550	F_CT_: 0.001	0.145
**Genetically based grouping (A and B)**						
**Between populations**	1	743.68	29.546	91.250	F_ST_: 0.912	0.000
**Within populations**	132	374.021	2.834	8.750		
**Total**						
**Between populations**	14	129.613	0.109	1.300	F_ST_: 0.013	0.284
**Within populations**	119	988.089	8.303	98.700		

Genetic structure results from the software STRUCTURE with a clear peak value of the ΔK statistic (S1 Fig) at K = 2 were in agreement with the existence of two groups within our samples (S2 Table).

In accordance with the network patterns (Table 3, Fig 2), neutrality tests and the mismatch distribution of the haplotypes of group ‘A’ supported the expansion theories (Fu *FS* = -25.914 P≤0.001; Tajima *D* = -2.606 P≤0.001; SSD = 0.414 P>0.05; Harpending’s raggedness index 0.010 P>0.05), whereas Fu *FS* and Tajima *D* for group ‘B’ were positive and not significant, indicating a non-expanding population.

**Table 3:** Values of neutrality tests (*Fs* and *D*) and mismatch analysis sums of squared deviation (*SSD*) and Harpending’s raggedness index for Eurasian Collared Dove mtDNA COI region sequences.

	Neutrality test		Mismatch	
Group	Tajima*D*	Fu-*F*_*S*_	*SSD*	*Harpending’s raggedness*
**A**	-2.606**	-25.914**	0.414	0.010
**B**	0.674	1.811	0.050	0.043
**All**	-1.566*	-6.399	0.010	0.007

*P≤0.05.

**P≤0.001.

As shown by S2 Fig, analysis of genetic structure in the studied populations revealed statistically significant positive autocorrelation among individuals of *S*. *decaocto* located up to 2000 km apart (r = 0.124; P = 0.001), suggesting that individuals of *S*. *decaocto* located within 2000 km of each other were more similar genetically than expected at random, whereas those individuals separated by greater distances were less similar than expected. The correlation value was considerably higher in the 1000 km class (r = 0.781; P = 0.001), then steeply declined, indicating that genetic structuring can be detected up to this distance.

## Discussion

Europe has been colonised by the Eurasian Collared Dove in less than a century. This remarkable achievement has attracted keen interest from researchers, although information on the genetic diversity and structure of the species has been scarce. In the present work we used only a female-specific marker, and analysed mtDNA COI region sequences from 152 samples (134 of our own samples and 18 from GenBank) covering a wide distribution range. High genetic diversity and two genetic structures without geographical localisation were detected. To our knowledge, similarly detailed studies on genetic diversity and structure have been very rare even in the case of other Columbidae species.

### Genetic diversity

The number of polymorphisms (171) and haplotypes (52) were high in the studied species, the European Collared Dove, which suggests population expansion [45], similarly to previous reports on other *Columbidae* species studied all over the world using different parts of mitochondrial DNA as markers [46–48]. For example, mtDNA cytochrome-b sequences of 95 European Turtle Doves (*Streptopelia turtur*) from Europe (Bulgaria, France, Germany, Greece, Italy, Malta, Spain and the United Kingdom) yielded 40 haplotypes [44]. The high haplotype and nucleotide diversities observed in our study (0.843±0.037 and 0.030, respectively) are also in agreement with data on other birds, including the Eurasian Black Cap (*Sylvia atricapilla*) [49], the Grey Jay (*Perisoreus canadensis*) [50], the Hazel Grouse (*Terastes bonasia*) [51], but contrary to those reported for the Shark-shinned Hawk (*Accipter striatus*) and the Great Blue Heron (*Ardea herodias*) [52]. A large number of new (47) and singleton (37) haplotypes were observed in our study. All of these high values were distributed homogeneously within each geographical region studied, suggesting that the population size of the species is large and expanding [53]. Certain invasive species have high genetic diversity and an enhanced ability to evolve when occupying novel regions [54]. Lee [55] stated that in the case of most species the success of invasion depends more on their ability to respond to natural selection than on physiological tolerance. We are aware that there is urgent demand for additional population genetic data for the purpose of controlling invasive species before they adapt to the local environment and additional invading occurs [56].

### Genetic structure

Our 134 sequenced animals together with all 18 mtDNA COI sequences obtained from GenBank were aligned in order to extend the geographical area studied. An NJ tree was constructed. The most frequent haplotype was Ht1, previously described in *S*. *decaocto* in the Netherlands [22]. The topology of the NJ and the phylogenetic tree were the first indication for the existence of two groups (‘A’ and ‘B’) among the detected haplotypes (Figs 2 and 3). In the case of group ‘A’, high haplotype (0.804±0.037) and low nucleotide diversity (0.006±0.003) values with a star-like haplotype network pattern (Fig 2) suggest fast expansion from an ancestral population with small effective population size (Ne) [45]. This structure may also occur due to contemporary gene flow, similarly to the migratory Sandhill Crane (*Grus canadensis*) [57], the Blue Manakin (*Chiroxiphia caudata*) [58], the Wood Grouse (*Tetrao urogallus*) [46] and the House Sparrow (*Passer domesticus*) [59]. In the case of group ‘B’ we did not find a dominant mtDNA haplotype, but a few low-frequency haplotypes and a large number of singletons were detected (Fig 2). However, our hypothesis for the existence of two genetic groups in *S*. *decaocto* was in agreement with the results of our analysis of population differentiation.

The AMOVA test clearly indicated that 91.25% of the genetic variation occurred between groups ‘A’ and ‘B’ (Table 2), which can suggest a strong and stable genetic difference among the individuals studied, similarly to the European Ground Squirrel (*Spermophilus citellus*) [60] and Berthelot's Pipit (*Anthus berthelotii*) [61]. However, a lack of genetic structure was detected in other avian species, like the House Sparrow (*Passer domesticus*) [62], the Red-legged Partridge (*Alectoris rufa*) [63] and the European Turtle Dove (*Streptopelia turtur*) [64]. A low level of genetic differentiation among populations was observed in the case of the House Sparrow (*Passer domesticus*) [62], the Galapagos Dove (*Zenaida galapagoensis*) [47] and the Red-headed Wood Pigeon (*Columba janthina nitens*) [65]. Geographically based isolation was not detected among the populations using AMOVA either, similarly to the Galapagos Dove (*Zenaida galapagoensis*) among the five Galapagos Islands [47], where no significant differentiation was observed either. Calderón et al. [64] did not detect any evidence of population genetic structure among three alternative flyways (from Western, Central and Eastern Europe to the south) used by European turtle doves during their spring and autumn journeys between Europe and Africa.

The presence of two groups was further verified by the results of the analysis using STRUCTURE (S1 Fig). In this study, we also performed Fu’s *FS* and Tajima’s *D* test, analysis for mismatch distribution to study the historical demographic expansions of *S*. *decaocto*, which could have an important role in the patterns of genetic variability. All tests and analysis supported our hypothesis about the demography history of the newly described groups ‘A’ and ‘B’, indicating the rapid and sudden expansion of group ‘A’. Similar results were found for the Chinese Egret (*Egretta eulophotes)* [66] and the Japanese Wood Pigeon (*Columba janthina*) [48].

Statistically significant positive autocorrelation suggested that individuals of *S*. *decaocto* located within 2000 km of each other were genetically more similar than expected at random, whereas those individuals separated by greater distances were less similar than expected. Other studies concluded that short-distance (<50 km) bird movements serving natal dispersal are typical of the Eurasian Collared Dove, however a 650-km dispersal distance is also observed in the species based on banding records [16, 54]. Nowadays global warming and human activities have a strong effect on the evolution and distribution of various species, especially on long-distance migratory birds [64, 67–70]. Although *Columbidae* are usually recognized as good flyers, potential dispersal associated with such capabilities cannot be observed in every case [71] in spite of the fact that long-distance dispersal birds have a significant impact on maintaining the genetic diversity of the species.

## Conclusions

Results from this study, based on mtDNA COI sequences, showed high genetic diversity, signs of global demographic expansion and two genetically–but not geographically–separated groups in Eurasian Collared Dove. Given that mtDNA variation in this work is highly structured genetically, a strong female natal philopatry is suggested. However these results are still not decisive, it is necessary to use nuclear data (microsatellite DNA) and more samples in further analysis.

## Supporting information

S1 Table List of *Streptopelia decaocto* specimens obtained for this study, extracted, sequenced and deposited in GenBank. (PDF)

S2 Table The Evanno table output showing maximum value of ΔK at K = 2. (DOCX)

S1 Fig The optimal number of genetic clusters inferred by STRUCTURE for our data set. Rate of change in the log probability (prob.) of data between successive runs of K (ΔK).
(TIF)

S2 Fig Spatial autocorrelation correlogram plots. The plot depicts results obtained from all geographic regions. The analysis considered geographic distances with even distance classes of 1000 km. Lines “U” and “L” represent the 95% confidence values of the null hypothesis (there is no structure), with “r” representing the correlation coefficient.
(TIF)
